# Nonconvulsive status epilepticus in patients with acute subarachnoid hemorrhage is associated with negative arterial spin labeling on peri-ictal magnetic resonance images

**DOI:** 10.1016/j.heliyon.2024.e24754

**Published:** 2024-01-14

**Authors:** Yoshiteru Tada, Toshitaka Fujihara, Izumi Yamaguchi, Masaaki Korai, Shu Sogabe, Mai Azumi, Eiji Shikata, Koji Bando, Kohei Nakajima, Kenji Shimada, Nobuaki Yamamoto, Hiroki Yamazaki, Yuishin Izumi, Masafumi Harada, Yasuhisa Kanematsu, Yasushi Takagi

**Affiliations:** a Epilepsy Center, Tokushima University Hospital, 3-18-15, Kuramoto-cho, Tokushima, Tokushima, 770-8503, Japan; b Department of Neurosurgery, Graduate School of Biomedical Sciences, University of Tokushima, 3-18-15, Kuramoto-cho, Tokushima, Tokushima, 770-8503, Japan; c Department of Neurology, Graduate School of Biomedical Sciences, University of Tokushima, 3-18-15, Kuramoto-cho, Tokushima, Tokushima, 770-8503, Japan; d Department of Radiology, Graduate School of Biomedical Sciences, University of Tokushima, 3-18-15, Kuramoto-cho, Tokushima, Tokushima, 770-8503, Japan

**Keywords:** Arterial spin labeling, Nonconvulsive status epilepticus, Subarachnoid hemorrhage

## Abstract

**Purpose:**

Non-convulsive status epilepticus (NCSE) is characterized by repetitive or continuous seizures without convulsions. Arterial spin labeling (ASL) is useful for assessing hyperperfusion due to neurovascular unit coupling in patients with NCSE; subarachnoid hemorrhage (SAH) impairs the neurovascular unit. We hypothesized that the sensitivity of ASL in detecting NCSE is low in patients with SAH during the acute phase.

**Methods:**

Based on ASL findings obtained within 48 h after the clinical suspicion of focal-onset NCSE, we divided 34 patients into ASL-negative (no hyperperfusion; n = 10) and ASL-positive (confirmed hyperperfusion; n = 24) groups. We further divided the two groups according to the NCSE etiology: patients who were diagnosed with NCSE within 14 days after SAH onset (acute SAH, n = 11) and patients with NCSE due to factors other acute SAH (n = 23) and compared their characteristics.

**Results:**

In 10 of the 34 patients (29.4 %) the ASL findings were normal. The rate of acute SAH was significantly higher in ASL-negative- (n = 8, 80.0 %) than ASL-positive patients (n = 3, 12.5 %). The rate of patients in aphasic status was significantly lower in ASL-negative patients (n = 1, 10 %) than in ASL-positive patients (n = 12, 50.0 %).

**Conclusion:**

Normal ASL findings alone should not be used to exclude a diagnosis of NCSE particularly in patients in the acute phase of SAH with deterioration or no improvement in consciousness.

## 1 Introduction

Status epilepticus (SE) occurs when the mechanisms responsible for seizure termination failure, or by the mechanisms that result in the abnormal prolongation of seizures are initiated (after time point t_1_). After time point t_2_, depending on the type and duration of the seizures, long-term consequences can develop. These include neuronal injury or death, and changes in neuronal networks [1].

Nonconvulsive SE (NCSE) is characterized as continuous nonconvulsive seizures that lasts more than 30 min or as repetitive nonconvulsive seizures over more than 30 min without complete recovery of sensory motor- and/or cognitive functions between successive attacks. The diagnosis of NCSE is based on electroencephalography (EEG) findings. The Salzburg Consensus Criteria (SCC) were formulated to improve the accuracy of an NCSE diagnosis [2,3].

Arterial spin labeling (ASL) is a repeatable and noninvasive perfusion imaging method which utilizes magnetically labeled water in the blood as an endogenous tracer [4]. ASL detects an increase in cerebral blood flow (CBF) in affected brain regions due to neurovascular unit coupling in the ictal and peri-ictal periods of SE and focal onset seizures [5,6].

Elsewhere [7] we reported cerebral hyperperfusion within 48 h of seizure onset in 33 of 41 patients (80.5 %) with focal seizures and noted that focal aware seizures were associated with normal ASL findings. Matsuura et al. [8] found that ASL recognized focal hyperperfusion in 13 of 20 patients with SE (65 %) in the peri-ictal state and Shimogawa et al. [9] documented ictal hyperperfusion in all 15 patients with NCSE, indicating that ASL is superior to of diffusion-weighted imaging (DWI).

In 3–15 % of patients with acute-phase aneurysmal subarachnoid hemorrhage (SAH) NCSE was observed [[10], [11], [12]]. As SAH impairs the neurovascular unit [13], we hypothesized that the sensitivity of ASL in the detection of NCSE is low in patients with SAH in the acute phase, examined the rate of ASL-negative findings in NCSE patients, and recorded the clinical characteristics and imaging findings of such patients.

## 2 Materials and methods

### 2.1 Patients

This study was approved by the Clinical Research Review Board of our institution (ethical approval number 3649). Informed written informed consent was obtained from all participants or their families involved in the study. We retrospectively evaluated 110 consecutive patients who were either admitted to our hospital with a clinical picture of seizure or subseqently diagnosed with seizures related to epilepsy or with acute symptomatic seizures between February 2016 and June 2022. Based on SCC, 42 patients were diagnosed with NCSE [2,3]. One was excluded due to generalized-onset NCSE. For 36 of the other 41 patients ASL images and EEG data were obtained within 48 h after the clinical suspicion of focal-onset NCSE; these patients were available for analysis. We then excluded another 2 patients from further data analyses owing to severe magnetic resonance imaging (MRI) artifacts. The remaining 34 patients [14 males, (41.2 %), 20 females (58.8 %), mean age 68.6 ± 16.8 years] were divided into ASL-negative (n = 10) and ASL-positive groups (n = 24) based on ASL findings. We then further divided members in these two groups according to the NCSE etiology: patients who were diagnosed with NCSE within 14 days of SAH onset (acute SAH, n = 11) and patients with NCSE attributed to factors other than acute SAH (n = 23). NCSE was classified using the extent of impaired awareness and whether NCSE occurred before or followed convulsive SE, as per the International League Against Epilepsy [1]. The aphasic status was included in the category of NCSE without coma and subclassified under focal SE [1]. EEG findings were categorized in association with NCSE using the proposed terminology [2,3,14], i.e:

(1) Epileptiform discharges, frequency more than 25/10-sec epoch
(2) Epileptiform discharges, frequency equal to or fewer than 2.5 cycles/sec or continuous (quasi) rhythmic delta activity, frequency more than 0.5 cycles/sec plus at least one of the following:
  (2a) Clinical and EEG improvement using i.v. antiepileptic agents
  (2b) Subtle clinical phenomena during EEG
  (2c) Typical spatiotemporal evolution
  (2d) EEG improvement with i.v. antiepileptic agent only
  (2e) Fluctuation in EEG findings in the absence of definitive evolution
(3) The absence of (1) or (2)

We categorized 1, and 2a-2c as NCSE, 2d-2e as possible NCSE, and 3 as not NCSE [2,3,14], and defined electrographic seizures by the presence of either rhythmic discharges or a spike-and-wave pattern of more than 10 s duration and having a definitive evolution in morphology, location, frequency, or amplitude [15].

For patients with acute SAH (n = 11), we recorded their Glasgow Coma Scale (GCS) on admission, their World Federation of Neurological Surgery (WFNS) grade, the presence of angiographic vasospasm at the time NCSE was suspected and during the acute phase of SAH, and the observation of delayed cerebral ischemia (DCI) when NCSE was suspected and during the acute phase of SAH. Vasospasm was evaluated using magnetic resonance angiography (MRA), digital subtraction angiography (DSA), or both, and characterized as a diffuse or segmental narrowing of greater than 30 % of the blood vessel diameter in large cerebral arteries vis-à-vis baseline measurements. DCI was recorded when new infarcts were seen on any follow-up radiological images obtained during the treatment course and diagnosed based on functional manifestations, i.e. clinical deterioration due to DCI upon the exclusion of any other potential inciting factor, including NCSE [16,17].

### 2.2 Imaging protocols

MRI scans were on a 3-T MRI scanner (Discovery MR 750; GE Healthcare, Milwaukee, WI, USA) with an 8-channel phased-array head coil. All 34 patients underwent DWI and ASL. Imaging sequences and parameters were DWI field of view (FOV) of 24 cm; matrix of 128 × 128; echo time (TE) of 65 ms; repetition time (TR) of 6000 ms; slice thickness of 5 mm; number of slices of 30; gap of 0 mm; b-factor of 1000; number of excitations (NEXs) of 2; and acceleration factor of 2. ASL images were acquired using a pseudo-continuous pulse sequence. Parameters were 512 sampling points on 8 spirals; FOV of 24 cm; reconstructed matrix, 64 × 64; TE of 10.5 ms; TR of 4632 ms; slice thickness, 4 mm; number of slices, 36; NEXs 2; and post-labeling delay (PLD) 2000 ms. Gray-scale CBF maps were generated according to Wang et al. [18].

### 2.3 Image analysis

All images were visually examined for hyperintensities on ASL and DWI data by two readers, M.H., a board-certified neuroradiologist and T.F., a neurosurgeon and board-certified epileptologist respectively with 31 and 17 years' experience blinded to clinical information and MRI data. The 2 observers, along with a 3rd and 4th reader inspected the images. The final decision was by consensus regarding positive or negative ASL and DWI findings. Positive signs were recorded based on consensus; when no unanimous decision was reached the sign was recorded as negative. Only the consensus judgments on ASL and DWI studies were used for further analysis; the individual observers’ judgments were used only for calculating inter-rater agreement.

### 2.4 Statistical analyses

Mean and standard deviations are shown for normally distributed variables and the median and interquartile range are shown for non-normally distributed variables. Normality was assessed using the Shapiro-Wilk test. Numeric, and nonparametric numeric variables were compared using the Fisher exact test, Student's *t*-test, and Mann-Whitney *U* test, respectively. Inter-rater agreement for T.F. and M.H. on the presence or absence of hyperintensity on ASL and DWI data was assessed with linear kappa (κ) coefficients. Statistical analyses were conducted using JMP version 13.2 (SAS Institute Inc., Cary, North Carolina, USA), with *p* < 0.05 considered to indicate statistical significance.

## 3 Results

### 3.1 Clinical characteristics

The clinical characteristics of the 34 NCSE are summarized in Table 1 and listed in Table 2, Table 3. A total of 29 patients (85.3 %) were diagnosed with NCSE and 5 (14.7 %) with possible NCSE based on EEG results and subtle clinical phenomena under the SCC. To detect electrographic seizures or to determine the required duration of drug treatments, 11 patients (32.4 %) underwent continuous video EEG monitoring for more than 24 h. Electrographic seizures were recorded in 4 of 11 patients (36.4 %). The interval between electrographic seizures and the acquisition of MRI scans was 20- (case 12), 8- (case 26), 3- (case 33), and 5 h (case 34). Of the 34 patients with NCSE, 3 (8.8 %) had no impairment of awareness and 31 (91.2 %) patients manifested mild to moderate impairment of awareness. Thirteen (38.2 %) presented with aphasia, and in 7 (20.6 %) we found prolonged awareness impairment after convulsive seizures.

**Table 1:** Clinical and radiological characteristics of ASL-negative and ASL positive NCSE patients (n = 34).

	Total (n = 34)	ASL-negative (n = 10)	ASL-positive (n = 24)	*P* value
Age, years, mean ± SD	68.6 ± 16.8	72.2 ± 22.2	67.1 ± 14.3	0.5130
Male, *n (%)*	14 (41.2 %)	2 (20.0 %)	12 (50.0 %)	0.1068
NCSE without impairment of awareness, *n (%)*	3 (8.8 %)	1 (10 %)	2 (8.3 %)	0.7995
Aphasic status, *n (%)*	13 (38.2 %)	1 (10 %)	12 (50.0 %)	0.0318*
NCSE with mild to moderate impairment of awareness, *n (%)*	31 (91.2 %)	9 (90 %)	22 (91.7 %)	0.6618
NCSE in coma, *n (%)*	5 (14.7 %)	1 (10 %)	4 (16.7 %)	0.5346
Convulsive status epilepticus preceding or succeeding NCSE, *n (%)*	7 (20.6 %)	0 (0 %)	7 (29.2 %)	0.0643
Etiology, *n (%)*				
Acute SAH	11 (32.3 %)	8 (80.0 %)	3 (12.5 %)	0.0003*
Other than acute SAH	23 (67.6 %)	2 (20.0 %)	21 (87.5 %)	
Rescue before MRI, *n (%)*	17 (50.0 %)	3 (30.0 %)	14 (58.3 %)	0.1294
Time from suspected NCSE to MRI, hours, median (IQR)	3.0 (1.0–12.5)	2.0 (0.5–12.0)	3.0 (1.9–10.3)	0.3052
DWI-positive findings, *n (%)*	13 (38.2 %)	0 (0 %)	13 (54.2 %)	0.0027*

ASL: arterial spin labeling, NCSE: nonconvulsive status epilepticus, SAH: subarachnoid hemorrhage, MRI: magnetic resonance imaging, DWI: diffusion-weighted imaging, SD: standard deviation, IQR: interquartile range.

*P < 0.05.

**Table 2:** Clinical profiles and MRI and EEG findings in 10 NCSE patients with normal ASL findings.

Case no.	Age (years)/sex	Etiology	Diagnosis of NCSE using the Salzburg criteria	Observed symptoms	Aphasic status	Time from suspected NCSE to MRI (hours)	EEG findings
**1**	81/M	Day 6 after SAH due to ruptured Rt. IC-PC aneurysm	2d	Coma	–	18	1.5–5 Hz generalized rhythmic delta/theta activity
**2**	72/F	Day 4 after SAH due to ruptured Lt. BA-SCA aneurysm	2a	Impaired awareness	–	0	1.0 Hz GPD
**3**	71/M	Day 13 after SAH due to ruptured Lt. ICA aneurysm	2a	Impaired awareness	–	48	2.0 Hz GRDA
**4**	12/F	Subacute phase after surgery for Rt. temporal glioma	2a	Impaired awareness	–	6	1.0 Hz bifrontal RDA
**5**	85/F	Day 2 after SAH due to ruptured Rt. IC-PC aneurysm	2a	Impaired awareness, hemispatial neglect	–	0.5	1.0–2.0 Hz LPD
**6**	79/F	Day 9 after SAH due to ruptured A-comA aneurysm	2b	Impaired awareness, limb myoclonus	–	0.5	1.0 Hz LPD
**7**	78/F	Day 9 after SAH due to ruptured Lt. ICA aneurysm	2d	Impaired awareness	–	1	0.5–5.0 Hz lateralized rhythmic theta-delta activity
**8**	92/F	Day 4 after SAH due to ruptured distal ACA aneurysm	2a	Impaired awareness	–	0.5	2.0 Hz bifrontal RDA
**9**	71/F	Day 9 after SAH due to ruptured A-comA aneurysm	2a	Impaired awareness, eye deviation, hemispatial neglect	–	3	2.0 Hz LPD
**10**	81/F	Epilepsy after head traumatic injury	2a	Aphasia	+	14	1.0–1.5 Hz Bifrontal RDA

MRI: magnetic resonance imaging, EEG: electroencephalography, ASL: arterial spin labeling, NCSE: nonconvulsive status epilepticus, DWI: diffusion-weighted imaging, M: male, F: female, Lt: left, Rt: right, SAH: subarachnoid hemorrhage, IC-PC: internal carotid-posterior communicating artery, BA-SCA: basilar artery-superior cerebellar artery, ICA: internal carotid artery, A-comA: anterior communicating artery, ACA: anterior cerebral artery, GPD: generalized periodic discharge, GRDA: generalized rhythmic delta activity, RDA: rhythmic delta activity, LPD: lateralized periodic discharge.

**Table 3:** Clinical profiles and MRI and EEG findings in 24 patients with ASL-positive findings.

Case no.	Age (years)/sex	Etiology	Diagnosis of NCSE using the Salzburg criteria	Observed symptoms	Aphasic status	Time from suspected NCSE to MRI (hours)	EEG findings
**11**	68/F	Old Rt. occipital infarction	2a, 2b	Impaired awareness, eye deviation, hemispatial neglect, Lt. hemiparesis	–	48	1.0 Hz LPD
**12**	56/M	Past history of surgery for Lt. putaminal hemorrhage	2c	Impaired awareness	+	1.5	Lt. centro-temporo-parietal rhythmic fast activity with evolution
**13**	47/F	Bilateral hippocampal sclerosis	2a, 2b	Impaired awareness, eye deviation	–	5	0.5–5.0 Hz GRDA
**14**	61/F	Day 6 after neck clipping for Rt. MCA unruptured aneurysm	2a	Aphasia	+	3	0.5–2.0 Hz LRDA
**15**	69/F	Day 6 after SAH due to ruptured Rt. MCA aneurysm	2b	Coma, eye deviation	–	17	2.0 Hz LPD
**16**	71/M	Subacute phase after surgery for Lt. chronic subdural hematoma	2a	Aphasia	+	1	1.5 Hz LRDA
**17**	79/M	Unknown	2b, 2c	Impaired awareness, eye deviation	–	30	Lt. centro-parietal rhythmic theta with evolution
**18**	75/M	Old Rt. temporal infarction	2a	Impaired awareness	–	1.5	1.5–2.0 Hz LRDA
**19**	83/M	Unknown	2c	Impaired awareness, cognitive impairment, aphasia	+	2	Lt. temporal rhythmic theta with evolution
**20**	75/M	Old Lt. temporal infarction	2d	Impaired awareness, aphasia, Rt. hemiparesis	+	3	1.0 Hz LPD
**21**	58/F	Past history of surgery for ruptured multiple aneurysms	2c	Coma	–	6	1.5–2.0 Hz LRDA
**22**	81/F	Day 2 after endovascular surgery for carotid cavernous fistula	2a	Impaired awareness, aphasia	+	3	1.0–2.0 Hz LPD
**23**	83/F	Day 5 after neck clipping for unruptured Rt. MCA aneurysm	2a, 2b	Impaired awareness, twiching of Lt. mouth	–	2	0.5–3 Hz LRDA
**24**	53/F	Metastatic brain tumor	2a	Coma	+	2	1.0–1.5 GPD
**25**	86/F	Acute phase of Lt. frontal cerebral hemorrhage	2a	Impaired awareness, aphasia, clonic seizure on Lt. face	+	48	1.0 Hz LPD
**26**	23/M	Day 4 after SAH due to ruptured Lt. ICA aneurysm	2c	Impaired awareness, limb myoclonus	–	3	1.0–2.0 Hz LRDA with evolution
**27**	60/M	Day 1 after neck clipping for unruptured A-comA aneurysm	2a	Impaired awareness	–	8	0.5–1.5 Hz GRDA
**28**	73/M	Rt. occipital malignant lymphoma	2a	Impaired awareness, myoclonus of Lt. upper limb	–	1	2.0–5.0 Hz lateralized rhythmic theta-delta activity
**29**	50/F	Past history of surgery for Rt. frontoparietal subcortical hemorrhage	2a, 2b	Impaired awareness, myoclonus of Lt. upper and lower limbs	–	2.5	1.0 Hz LPD
**30**	71/M	Old Lt. parietal hemorrhage due to arteriovenous malformation	2b	Impaired awareness, eye deviation	+	48	1.0 Hz LPD
**31**	78/F	Day 8 after SAH due to ruptured A-com aneurysm	2d	Impaired awareness, aphasia	+	0.5	1.5 Hz LRDA
**32**	75/F	Lt. temporal metastatic brain tumor	2d	Impaired awareness, aphasia	+	20	1.5 Hz LRDA
**33**	69/M	Day 4 after surgery for craniopharyngioma	2b, 2c	Impaired awareness, eye deviation	–	1	1.0 Hz LPD
**34**	66/M	Occipital lobe epilepsy	2c	Impaired awareness, aphasia, homonymous hemianopsia	+	2	Lt. occipital rhythmic theta with evolution

MRI: magnetic resonance imaging, EEG: electroencephalography, ASL: arterial spin labeling, NCSE: nonconvulsive status epilepticus, DWI: diffusion-weighted imaging, M: male, F: female, Lt: left, Rt: right, MCA: middle cerebral artery, SAH: subarachnoid hemorrhage, ICA: internal carotid artery, A-comA: anterior communicating artery, LPD: lateralized periodic discharge, GRDA: generalized rhythmic delta activity, LRDA: lateralized rhythmic delta activity, GPD: generalized periodic discharge.

The 34 patients were classified into two groups by NCSE etiology; 11 (32.4 %) presented with acute SAH (n = 11) in 23 (67.6 %) factors other than acute SAH were involved. Before undergoing MRI, 17 patients (50 %) had received rescue medications. The median interval between suspecting NCSE and the acquisition of MRI scans was 3.0 h (interquartile range, 1.0–12.5 h). The inter-rater agreement for T.F. and M.H. on the presence or absence of hyperintensity on ASL and DWI studies was good (κ = 0.91 and κ = 0.88, respectively). They detected high-intensity lesions on DWI scans of 13 patients (38.2 %).

### 3.2 Representative cases

#### 3.2.1 Case 2

In this 72-year-old woman with NCSE, ASL findings were negative during acute SAH (Fig. 1A). A left basilar artery-superior cerebellar aneurysm had ruptured and she underwent coil embolization. On the 4th day thereafter her Glasgow Coma Scale (GCS) score fell to 6, she underwent emergency MRI. ASL and DWI findings revealed no abnormalities (Fig. 1B and C). MRA denied vasospasm (Fig. 1D). EEG performed 12 h after GCS deterioration revealed 1.0 Hz generalized periodic discharges (GPD) (Fig. 1E). After the administration of midazolam and lacosamide there was marked EEG improvement. On the 8th post-embolization day her consciousness gradually recovered to GCS score of 9 and she was diagnosed with NCSE.

**Fig. 1:** Imaging and EEG findings. Computed tomography showing SAH (A). ASL revealed no hyperintense lesions (B). DWI also showed no hyperintense lesions (C). MRA denied vasospasm (D). EEG recording presented as a longitudinal bipolar montage shows 1.0 Hz generalized periodic discharge (E).

#### 3.2.2 Case 29

A 50-year-old woman with a history of surgery for right frontoparietal subcortical hemorrhage due to Moyamoya disease. She presented with generalized convulsions. Her generalized convulsive seizures were maintained under control with fosphenytoin sodium and levetiracetam. However, her GCS 24 h after their administration remained 5. There was myoclonus on the left side of the upper and lower limbs. ASL revealed hyperperfusion in the right fronto-temporo-occipital cortex (Fig. 2A and B). There were no abnormalities on DWI scans (Fig. 2C and D). EEG revealed 1.0 Hz lateralized periodic discharges at the right hemisphere (Fig. 2E). One day after the administration of midazolam and lacosamide, the EEG results improved notably; her score on the GCS was 14 and her myoclonus disappeared a day later.

**Fig. 2:** Imaging and EEG findings. Hyperintensity on the ASL image of a 50-year-old woman with NCSE. (A and B) Note the hyperintensity area on ASL in the right fronto-temporo-occipital cortex (arrowheads). (C and D) DWI reveals no lesions. (E) EEG recording presented as a longitudinal bipolar montage shows 1.0 Hz lateralized periodic discharges at the right hemisphere (square).

### 3.3 Factors associated with ASL-negative findings in patients with NCSE

ASL findings were normal in 10 of our 34 patients (29.4 %); they showed focal hyperintensity in 24 (70.6 %). Table 1 compares the radiological and clinical characteristics of ASL-negative and ASL-positive patients. The rate of acute SAH was significantly increased among ASL-negative- compared with ASL-positive patients (8/10, 80.0 % vs 3/24, 12.5 %, respectively, *p = 0.0003*). ASL findings were normal in 8 of 11 patients with acute SAH (72.7 %); in 21 of 23 patients (91.3 %) with inciting factors other than acute SAH, ASL demonstrated hyperintensity.

The rate of aphasic status was significantly lower among ASL-negative- (1/10, 10 %) than ASL-positive patients (12/24, 50 %); *p = 0.0318*. We found no significant inter-group differences in the NCSE patients’ mean age and sex, the administration of rescue medications before MRI, the median interval between the time NCSE was suspected and the acquisition of MRI scans, the number of patients without- or with mild to moderate awareness, and the number of NCSE in coma. A trend toward a lower prevalence of convulsive SE preceding or succeeding NCSE was seen in the ASL-negative group compared to that in the ASL-positive group (0 % vs. 29.2 %), albeit without statistical significant. DWI findings were positive only in ASL-positive patients; the inter-group difference was significant (*p* = 0.0027).

### 3.4 Clinical characteristics of patients with acute SAH

NCSE was diagnosed in 11 patients (4 males (36.4 %), 7 females (63.6 %), mean age 72.6 ± 17.8 years) during the acute phase of SAH. Clinical characteristics are summarized in Table 4. The WFNS grade was 4–5 of the 11 patients (45.5 %). When NCSE was suspected, in one of these patients (9.1 %) we detected angiographic vasospasm and DCI; the ASL finding were normal. In contrast, 4 (36.4 %) and 6 (54.5 %) of the 11 patients had angiographic vasospasm and DCI during the acute phase of SAH, respectively. Therefore, NCSE seems to precede vasospasm and DCI.

**Table 4:** Clinical profiles of 11 patients with acute SAH.

Case no.	Age (years)/sex	ASL findings	GCS score at admission	WFNS grade	Angiographic vasospasm at suspicion of NCSE	Angiographic vasospasm during acute phase of SAH	DCI at suspicion of NCSE	DCI during acute phase of SAH
**1**	81/M	Negative	13	2	–	–	–	–
**2**	72/F	Negative	14	2	–	–	–	–
**3**	71/M	Negative	13	2	–	+	–	+
**5**	85/F	Negative	15	1	–	–	–	–
**6**	79/F	Negative	12	4	+	+	+	+
**7**	78/F	Negative	10	4	–	+	–	+
**8**	92/F	Negative	15	1	–	–	–	–
**9**	71/F	Negative	9	4	–	–	–	+
**15**	69/F	Positive	7	5	–	–	–	+
**26**	23/M	Positive	4	5	–	+	–	+
**31**	78/F	Positive	15	1	–	–	–	–

ASL: arterial spin labeling, GCS: Glasgow Coma Scale, WFNS: World Federation of Neurological Surgery, NCSE: nonconvulsive status epilepticus, SAH: subarachnoid hemorrhage, DCI: delayed cerebral ischemia, M: male, F: female.

## 4 Discussion

Here, we retrospectively compared clinical and imaging findings associated with ASL-positive and ASL-negative findings in patients with NCSE. We found a probability of false-negative findings on pseudo-continuous ASL imaging with a PLD of 2.0 s using a 3-T MRI of 29.4 %, and a low sensitivity of ASL in detecting NCSE in the acute phase of SAH of 27.3 %.

During seizures, cerebral metabolic demands rapidly increase and the regional CBF increases [19]. Because ASL can detect the perfusion increase due to neurovascular unit coupling as a result of the seizure activity, it is useful for detecting hyperperfusion in patients with SE and NCSE [6,8,9,14]. In patients with SE, hyperperfusion was detect by ASL in 13 of 20 patients (65 %) and in 42/46 (91.3 %) [6,8]. In patients with NCSE, hyperperfusion was detected in 15 of 15 patients (100 %) and in 24 of 24 episodes [9,14]. Others [6,8] found that ASL was superior to DWI with respected to the identification of SE and NCSE.

We obtained ASL-negative findings in 10 of 34 (29.4 %) patients. Acute SAH was associated with normal ASL findings; the ASL-positive rate was high (91.3 %) among patients with NCSE due to factors other than acute SAH. Diseases including brain tumors, arteriovenous malformation, Moya Moya disease, and cerebral infarction impair the neurovascular unit, however, they result in relatively focal damage. On the other hand, as SAH impairs the neurovascular unit diffusely [13], we hypothesized that such impairment avoids hyperperfusion during the acute SAH phase. Alternatively, post-SAH vasospasm may reduce the CBF and avoid a CBF increase in NCSE patients. However, angiographic vasospasm and DCI were observed in only one of our 11 patients (9.1 %) with acute SAH at the time we suspected NCSE. Prospective studies on larger populations of NCSE patients are required to investigate the relationship between ASL findings and the presence of vasospasm and DCI. In NCSE patients, induced hypertension to address post-SAH DCI may increase the CBF and affect the ASL findings, however, we did not induce hypertension in our patients with SAH. NCSE or SE was reported in in 3–15 % of patients with aneurysmal SAH during the acute phase [[10], [11], [12]]. NCSE and SE may contribute to the severe secondary brain damage associated with neurocognitive and neurological deficits [[10], [11], [12]]. Consequently, an early diagnosis and treatment are required. Although NCSE in addition to vasospasm during the acute period of SAH should be diagnosed, the rate of false-negative findings on ASL is relatively high, especially in patients with acute SAH.

Among our 34 patients we performed continuous video EEG monitoring (more than 24 h) in 11 patients (32.4 %) to detect electrographic seizures or to determine the required duration of drug treatments. Electrographic seizures were recorded in 4 of 11 patients (36.5 %). Kim et al. [6] who also performed continuous EEG and ASL identified hyperperfusion in 42 of 51 SE patients (82.4 %). Shimogawa et al. [9] diagnosed NCSE based on their initial MRI findings followed by routine EEG; ASL identified hyperperfusion in all of their 15 patients. Ohtomo et al. [14] recorded cortical hyperperfusion in all of 21 episodes suffered by patients with NCSE or possible NCSE; 12 of the episodes were recorded under continuous EEG monitoring exceeding 6hr. We suspect that short-term EEG recordings may miss informative epochs. Differences in the approaches applied by diagnosticians approach may explain differences in the identification of hyperperfusion by ASL. Elsewhere [7] we reported that the MRI technique also may affect the detection of hyperperfusion on ASL data.

The aphasic status is a subtype of focal NCSE [1], and its accurate diagnosis is important for adequate treatment. Although others [20,21] reported that ASL revealed hyperperfusion in patients with aphasic status, its diagnostic value of in such patients requires further evaluation. We excluded patients with diseases such as cerebral infarction, cerebral hemorrhage, and/or brain edema because they show aphasia on MRI scans including DWI, ASL-, T2* weighted imaging-, and MRA scans. Our diagnosis of the aphasic status based on Salzburg consensus criteria. In all patients of our 13 patients with aphasia it was improved by treatment with antiepileptic drugs; 12 of 13 patients (92.3 %) were ASL positive and only one was ASL-negative (p < 0.0318). Although ASL might be useful to diagnose aphasic status, further studies with a larger number of patients are required.

Several limitations of our study warrant mention. First, it was conducted retrospectively and included a relatively small number of enrolled patients. Therefore, further studies with a larger number of patients are required. Second, some of our not NCSE patients did not undego both ASL and DWI imaging during the study period. Occasionally, it was difficult to perform MRI for patients with NCSE in coma who required artificial respiration. Consequently, we cannot deny selection bias. Third, we acknowledge that before suspecting NCSE and in the interval between suspected NCSE and acquiring MRI scans, NCSE may have been present and may have been resolving. Lastly, some NCSE patients did not undergo continuous EEG during the study period.

In conclusion, our findings suggest that normal ASL findings alone should not be used to exclude a diagnosis of NCSE, particularly in patients in the acute phase of SAH with deterioration or no improvement in consciousness. We propose that NCSE diagnosis should be based on a combination of clinical symptoms and MRI and EEG findings.

## Institutional review board statement

This study was approved by the Clinical Research Review Board of our institution (ethical approval number 3649).

## Funding

This study received no funding from public, commercial, or not-for-profit organizations.

## Date availability statement

Data will be made available on request.

## CRediT authorship contribution statement

**Yoshiteru Tada:** Writing - review & editing, Writing - original draft, Validation, Methodology, Investigation, Formal analysis, Data curation, Conceptualization. **Toshitaka Fujihara:** Validation, Investigation, Formal analysis, Data curation. **Izumi Yamaguchi:** Validation, Investigation, Formal analysis, Data curation. **Masaaki Korai:** Validation, Investigation, Formal analysis, Data curation. **Shu Sogabe:** Validation, Investigation, Formal analysis, Data curation. **Mai Azumi:** Validation, Investigation, Formal analysis, Data curation. **Eiji Shikata:** Formal analysis, Data curation. **Koji Bando:** Validation, Investigation, Formal analysis, Data curation. **Kohei Nakajima:** Validation, Investigation, Formal analysis, Data curation. **Kenji Shimada:** Validation, Investigation, Formal analysis, Data curation. **Nobuaki Yamamoto:** Validation, Investigation, Formal analysis, Data curation. **Hiroki Yamazaki:** Validation, Investigation, Formal analysis, Data curation. **Yuishin Izumi:** Validation, Investigation, Formal analysis, Data curation. **Masafumi Harada:** Validation, Investigation, Formal analysis, Data curation. **Yasuhisa Kanematsu:** Validation, Investigation, Formal analysis, Data curation. **Yasushi Takagi:** Writing - review & editing, Writing - original draft, Validation, Supervision, Methodology, Investigation, Formal analysis, Data curation, Conceptualization.

## Declaration of competing interest

The authors declare that they have no known competing financial interests or personal relationships that could have appeared to influence the work reported in this paper.
